# An Improved Particle Swarm Optimization Algorithm and Its Application to the Extreme Value Optimization Problem of Multivariable Function

**DOI:** 10.1155/2022/1935272

**Published:** 2022-05-13

**Authors:** Min Cai

**Affiliations:** School of Mathematical and Statistics, Xuzhou University of Technology, Xuzhou 221008, China

## Abstract

It is proposed to improve the study of particle optimization and its application in order to solve the problem of inefficiency and lack of local optimization skills in the use of particle herd optimization. Firstly, the basic principle, mathematical description, algorithm parameters, and flow of the original (Particle Swarm Optimization, PSO) algorithm are introduced, and then the standard PSO algorithm is introduced; thirdly, over the last 10 years, four types of improvements have been proposed through the study of improved particle algorithms. The improved algorithm is applied to the extreme value optimization problem of multivariable function. The simulation results show that the basic (Cloud Particle Swarm Optimization, CPSO) algorithm within 500 generations has not reached convergence for 8 times, 6 times, 4 times, and 5 times, respectively. In the case of convergence, the average number of steps is much higher than ICPSO, and the improved algorithm converges completely. In terms of time performance, the convergence time of ICPSO is much better than that of CPSO algorithm. Therefore, the improved particle optimization algorithm ensures the effectiveness of the improvement measures, such as small optimization algebra, fast merging speed, high efficiency, and good population diversity.

## 1. Introduction

An optimization problem involves finding a set of parameter values under certain constraints so that some measure of optimization is met, even if some performance indexes of the system reach the minimum or maximum. It is an ancient subject based on mathematics. It widely exists in agriculture, chemical industry, national defense, finance, transportation, electric power, communication, and many other fields [1]. The application of optimization technology in the above fields has brought great economic and social benefits. Long-term practice shows that under the same conditions, the treatment of optimization technology has significant effects on the reduction of system energy consumption, the improvement of efficiency, and the rational utilization of resources, and this advantage is more obvious with the increase of the scale of treatment objects. The emergence of bionic algorithm provides a powerful tool for a large number of problems that cannot be well optimized by traditional optimization algorithms. Bionic algorithm is an algorithm model based on human and biological behavior or material movement form [2]. Since this kind of algorithm was put forward, because of its universality in solving the optimization problem, it does not need some information of the objective function or even the explicit expression of the optimized object. It only needs to know the input and output of the optimized problem so as to avoid the computational complexity and difficult operability of the algorithm based on the properties of the optimized function. Currently, bionic algorithms include genetic algorithms, artificial immunity algorithms, ant colony optimization algorithms, particle herd optimization algorithms, community location algorithms, and more [3, 4].

Particle swarm optimization (PSO) is a new type of bionic optimization algorithm that is similar to the genetic algorithm and is a repetitive optimization algorithm (see Figure 1). It initiates a set of random solutions and repeatedly searches for the optimal solution. However, this is different from the evolutionary idea in the genetic algorithm that “the best survives, the best survives.” Compared to other bionic algorithms, such as genetic algorithms, particle herd algorithms are simpler to understand, have fewer parameters that can be adjusted, and are easier to implement. Convergence analysis of particle herd optimization algorithms is the basis of PSO algorithms. Currently, most improved particle herd optimization algorithms lack convergence models and convergence analysis. Second, the particle optimization algorithm is easy to get into the local optimization problem; that is, there is a problem of incomplete integration [5]. Particle optimization when solving the problem of optimizing high-dimensional or ultra-high-dimensional complex functions, particle swarm optimization often has the problem of premature convergence; that is, limited by the particle update mechanism, the particles have gathered to a point and stagnated when the population has not found the optimal solution. Therefore, it is urgent to find an effective mechanism to make the algorithm escape from local minima and overcome the problem of premature convergence. Third, it is necessary to expand the theory of discrete particle optimization and its application, as the results of discrete particle optimization studies lag far behind continuous particle optimization. Fourth, the expansion of research on the application of particle herd algorithms, how to use particle herd algorithms, and the integration of other algorithms to solve practical problems are the research topics of domestic and foreign scientists [6].

## 2. Literature Review

Numerous scientists are devoted to the study of optimization problems, and as a result, optimization theories and algorithms are developing rapidly. Currently, traditional optimization methods include Newton's method, simplex method, and conjugate gradient method, trust region method, pattern search method, Rosenbrock method, and Powell method. When facing some large-scale problems, these methods need to traverse the whole search space and produce a combination explosion of search, which makes them “helpless” in the face of these problems; that is, the calculation speed, convergence, and initial sensitivity are far from meeting the requirements. Therefore, efficient optimization algorithm has become one of the research objectives of scientists [7]. Sun et al.'s model has been proposed to convert uncertainty between the definition of qualitative knowledge, the concept of quality, and its numerical representation, and it has been used in many fields, such as intelligent management and fuzzy evaluation. Because the cloud model has the characteristics of uncertainty, uncertainty, stability, and change in the expression of knowledge, it reflects the basic principles of species evolution in nature. Therefore, the field of evolutionary computing has also begun to focus on cloud design [8]. Song's algorithm for high-dimensional functions and nonlinear distribution particle optimization has been proposed to overcome the poor performance of particle optimization. The algorithm performs scattering operations on particles in a nonlinear increment so that a large number of unnecessary scattering operations can be avoided at the beginning of the algorithm iteration, and the probability of scattering operations at the end is high iteration, thus ensuring the efficiency of the algorithm's operation. This can effectively improve the algorithm's global search capability [9]. Zeng et al. proposed a cloud genetic algorithm by using cloud generator to replace the traditional crossover and mutation operators in genetic algorithm, which has achieved good results in function optimization [10]. Kumari et al. combining genetic algorithms with cloud models offers a cloud-based evolutionary algorithm that effectively solves the problem of genetic algorithms and easily facilitates local optimization and early convergence [11]. Omidinasab and Goodarzimehr proposed an adaptive cloud particle swarm optimization algorithm using particle fitness and different inertia weight evolution strategies, which effectively solved the problems of local optimization and too fast convergence speed of the algorithm [12]. Zhu et al. suggest that the current condition and space of a particle in an entire population should be explored, evaluated by the fitness value of the particle, and its speed adjusted by the fitness value so that the particle itself can be active locally and globally search [13].

Based on this study, this paper proposes to improve the study of particle herd algorithms and their applications. By means of solution space transformation, the local optimization and global optimization are combined, a simple cloud operator is used to study the evolution of particles and to perform mutations to accelerate the integration speed of the algorithm. From the simulation results, it can be seen that the improvement measures improve the accuracy of the population diversity, search capabilities, and algorithm integrity.

## 3. Research Methods

### 3.1. Particle Herd Algorithm

Particle herd optimization (PSO) is a new type of bionic optimization algorithm based on modeling the behavior of birds of prey according to certain assumptions. The discovery of the algorithm is based on the modeling of simplified social models. It originated from complex adaptive system. CAS particle swarm optimization algorithm is developed based on the following four characteristics of CAS: firstly, the subject is active and active. Secondly, the subject interacts with the environment and other subjects, which is the main driving force for the development and change of the system. Moreover, the influence of environment is macro, the influence between subjects is micro, and macro and micro should be organically combined. Finally, the whole system may also be affected by some random factors [14].

#### 3.1.1. Standard Particle Swarm Optimization Algorithm

In order to better explore the solution space, Shi introduced the concept of inertia weight based on the original particle herd algorithm and gradually developed the standard particle herd algorithm currently in use. The speed-position update mode is as follows:

(1) $$\begin{array}{c} v_{i}^{j+1}=\omega v_{i}^{j}+c_{1}\xi \left(p_{i}^{j}-x_{i}^{j}\right)+c_{2}\eta \left(p_{g}^{j}-x_{i}^{j}\right), \end{array}$$

(2) $$\begin{array}{c} x_{i}^{j+1}=x_{i}^{j}+v_{i}^{j+1}. \end{array}$$

The standard particle herd algorithm described in this section is a linearly tuned particle herd algorithm. Its formula is

(3) $$\begin{array}{c} \omega =\left(\omega_{\max}-\omega_{\min}\right)\left(\frac{\text{Gen}-\text{iter}}{\text{Gen}}\right)+\omega_{\min}, \end{array}$$

where *ω*_max_ indicates the value of the maximum mass of inertia, *ω*_min_ indicates the minimum value of the mass of inertia, Gen represents the maximum number of iterations, and iter represents the current number of iterations. A particle herd algorithm involves inertial motion of a particle along its own velocity and thinking about the behavior of the particle itself. At the same time, it also participates in group information sharing and mutual cooperation so as to find the best position in the particle swarm. The interaction and restriction of these three parts determine the optimization performance of the algorithm [15, 16]. For its movement process, see Figure 2.

#### 3.1.2. Discrete Particle Swarm Optimization

To solve the problem of optimizing a separate combinator with a PSO algorithm, two completely different technical routes were developed: one based on the classical continuous particle herd algorithm, and for a specific problem, a discrete policy space for continuous particle motion, space, and appropriate adjustments is made. The PSO algorithm to be solved still retains the speed-position update algorithm of the classical particle herd algorithm in the calculation. His representative, Eberhart, proposed a discrete binary version of the PSO based on the first particle herd algorithm. The model they proposed is to limit the historical and global optimization of each dimension of the particle and the particle itself to 1 or 0, but the speed is not limited. When updating the position with speed, set an off value. When the speed is higher than the off value, the position of particles is taken as 1; otherwise, it is taken as 0. The speed and position update equations are expressed as follows:

(4) $$\begin{array}{c} v_{id}^{j+1}=\omega v_{id}^{j}+c_{1}\xi \left(p_{id}^{j}-x_{id}^{j}\right)+c_{2}\eta \left(p_{gd}^{j}-x_{id}^{j}\right). \end{array}$$

(5) $$\begin{array}{c} \text{If}\left(r\text{ and}\left(\right)<S\left(v_{id}\right)\right)\text{, then }x_{id}=1, \end{array}$$

(6) $$\begin{array}{c} \text{Else }x_{id}=0. \end{array}$$

Consider

(7) $$\begin{array}{c} S\left(v_{id}\right)=\frac{1}{1+\exp\left(-v_{id}\right)}, \end{array}$$

where *S*(*v*_*id*_) is the sigmoid function and *r* and () is the random number between [0, 1]. The velocity component *v*_*id*_ determines the probability that the position component *x*_*id*_ takes 1 or 0. The greater the *v*_*id*_, the greater the probability that *x*_*id*_ takes 1.

Another approach is to solve the discrete optimization problem based on the basic information update mechanism of the PSO algorithm, as well as to redefine the basic idea of the classical particle optimization algorithm, the unique representation of the particle herd, and the operation algorithm within the algorithm, for example, the discrete binary PSO algorithm proposed by Farzane in Clerc's Traveler Trading Policy (TSP) and the 0–1 planning policy. The difference between the two methods lies in the following: the former maps the actual discrete problem to the particle continuous motion space and then calculates and solves it in the continuous space. The latter is to map PSO algorithm to discrete space and calculate and solve it in discrete space [17, 18].

### 3.2. Improved Particle Swarm Optimization (ICPSO)

#### 3.2.1. Cloud Design

The cloud model is a mathematical model that transforms deterministic knowledge into qualitative and quantitative forms and mainly reflects the ambiguity and randomness of knowledge about things and people in the objective world and provides a combination of qualitative and quantitative processing of things.

**Definition 1 .**

(clouds and cloud drops). Let *U* be a numerical world represented by numerical values, and *C* be a qualitative concept over *U*. If the numerical value of *x* ∈ *U* is a random embodiment of the concept of quality *C*, then *C µ* (*x*) ∈ [0, 1] of the degree of certainty is a random number that tends to be constant: *μ* : ∪⟶[0,1],  *x* ∈ ∪, *x*⟶*μ*(*x*). The distribution of *x* in the *U* universe is then called a cloud, which is denoted by a *C* (*X*) cloud, and each *x* is called a cloud drop. The cloud model and its numerical properties are shown in Figure 3, and *Ex* = 20, *En* = 3, *He* = 0.1.

**Definition 2 .**

One-dimensional simple cloud operator ArForward (*C* (*Ex*, *En*, *He*)) is a mapping of *π* that converts the general properties of quality concepts into digital representations. C ⟶Π. The following conditions are met:

(8) $$\begin{array}{c} \Theta =\left\{t_{i}|\text{Norm}\left(En,He\right),\;i=1,\cdots ,N\right\}.\\ X=\left\{x_{i}|x_{i},t_{i}\in \Theta ,\;i=1,\cdots ,N\right\}.\\ \prod =\left\{\left(x_{i},y_{i}\right)|x_{i}\in X,\;t_{i}\in \Theta ,\;y_{i}=\exp\left(-{\left(x_{i}-Ex\right)}^{2}/\left(2t_{i}^{2}\right)\right)\right\}. \end{array}$$

In, Norm(*μ*, *δ*) is a normal random variable with expected value *µ* and variance *δ*, and *N* is the number of cloud droplets. Using a simple cloud operator, it is possible to convert a concept into a set of cloud droplets numerically represented by *C* (*Ex*, *En*, *He*) realizing the transformation from conceptual space to numerical space. The one-dimensional simple cloud operator can be extended to the *n*-dimensional simple cloud operator.

#### 3.2.2. Basic Particle Swarm Optimization (CPSO)

Let the size of the particle swarm be *N*, the fitness value of the particle *X*_*i*_ in the *t*th iteration is *f*_*i*_, and the average fitness value of the particle is equations (8)∼(10):

(9) $$\begin{array}{c} f_{\text{avg}}=\frac{1}{N}\sum_{i=1}^{N}f_{i}, \end{array}$$

(10) $$\begin{array}{c} \upsilon_{id}^{\left(t\right)}=\omega \upsilon_{id}^{\left(t\right)}+c_{1}r_{1}\left(P_{id}-x_{id}^{\left(t\right)}\right)+c_{2}r_{2}\left(P_{gd}-x_{id}^{\left(t\right)}\right), \end{array}$$

(11) $$\begin{array}{c} x_{id}^{\left(t+1\right)}=x_{id}^{\left(t\right)}+\upsilon_{id}^{\left(t+1\right)}. \end{array}$$

Equations (9) and (10) are speed update formula and position update formula, respectively. The fitness value better than *f*_avg_ is averaged to get *f*_avg_′, the fitness value less than *f*_avg_ is averaged to get *f*_avg_^″^, and the fitness value of the optimal particle is *f*_min_. If *f*_*i*_ is better than *f*_avg_′, the fitness value of particles is small and close to the optimal solution. Small inertia weight is adopted, and the evolution strategy adopts “social model” to speed up the speed of global convergence. If *f*_*i*_ is inferior to *f*_avg_^″^, the fitness value of particles is large and far from the optimal solution. Large inertia weight is adopted, and the evolution strategy adopts “cognitive model” so that these particles with poor performance can accelerate the convergence speed. If *f*_*i*_ is better than *f*_avg_^″^ and inferior to *f*_avg_′, the fitness value of particles is moderate, the inertia weight adopts cloud adaptive inertia weight, and the evolution strategy adopts “complete model” [19].

**Definition 3 .**

(evolutionary model). The process that each particle generates a new generation of particles through the normal cloud generator according to its individual extreme value is called evolutionary model.

**Definition 4 .**

(mutation). Given the thresholds *N* and *K* in advance, when the global extreme value has not evolved for *N* consecutive generations or the amplitude of the evolution process is less than *k*, it is considered that the particles fall into the local optimum, and all particles are mutated through the normal cloud generator according to the global extreme value.

#### 3.2.3. ICPSO Algorithm

Aiming at the problems of the above basic CPSO, this paper puts forward the following two improvement methods.

(1) With the help of group substitution and spatial transformation, the global search and local search are combined.
Most of the running time of the basic CPSO algorithm is consumed in the updating of the population. In addition, the limitation of slow evolution often appears in the later stage of evolution. For this, group substitution and space transformation are introduced. The particle swarm optimization algorithm of group substitution mainly searches the solution space through several particle swarm optimization using different search methods. One particle swarm is the main search group and the other is the auxiliary search group. Under some conditions in the search process, some auxiliary search group particles and main search group particles are replaced to maintain the diversity of main search group particles so that the main search group can avoid stagnation or premature due to lack of diversity so as to ensure that the main search group can search the global optimal value point. In order to calculate the advantages and disadvantages of the current position of cloud particles, it is necessary to transform the solution space and map the two positions occupied by each particle from the unit space *I*=[−1,1]^*n*^ to the solution space of the optimization problem. Note that the *i*th cloud operator on particle *P*_*j*_ is [*α*_*i*_^*j*^*β*_*i*_^*j*^]^*T*^; then, the corresponding solution space variables are as follows:
  (12) $$\begin{array}{c} X_{k}^{j}=\frac{1}{2}\left[b_{i}\left(1+\alpha_{i}^{j}\right)+a_{i}\left(1-\alpha_{i}^{j}\right)\right], \end{array}$$
  (13) $$\begin{array}{c} X_{i\delta }^{j}=\frac{1}{2}\left[b_{i}\left(1+\beta_{i}^{j}\right)+a_{i}\left(1-\beta_{i}^{j}\right)\right]. \end{array}$$
Then, if the optimal value obtained is greater than the modern optimal solution, the spatial transformation of the solution is optimized. After each iteration, the improved algorithm performs local search near the contemporary optimal solution and improves the ability to search algorithms, and the basic CPSO algorithm improves errors that do not change over several generations [20].
(2) According to a simple cloud operator, particle mutations are used to improve the algorithmic search method. Nonmodern optimal solutions focus on phenomena that are common in the evolutionary process of the CPSO basic algorithm, and the greater the evolution, the greater the deviation from the optimal solution, and the following improvement measures are taken: calculate the initial value of the current position and velocity of each particle, and then calculate whether the fitness of each particle has reached the mutation threshold *N*, and if so, perform a mutation operation on each particle according to Definition 4; otherwise, the particle renewal is performed according to equations (9) and (10).

#### 3.2.4. Algorithm Flow of ICPSO

The ICPSO algorithm flow using the above two improvement measures is as follows:

1. Initialize the population. That is, initialize the position of each particle, individual extreme value PBEST, local extreme value GBEST, and so on.
2. Calculate the fitness value for each particle and update Pbest and Gbest.
3. Judge whether the mutation threshold *n* is reached. If it is reached, the mutation operation is carried out according to Definition 4. Let the local best (minimum) of all particles be Gbest and make *ex* = Gbest, *en* = 2gbest, *h*e = en/10 in normal cloud computing a (*C* (*ex*, *en*, *he*)). According to Definition 2, the normal cloud generator completes the mutation operation of all particles and fails to reach the mutation threshold (4).
4. Evolve each particle. Let the individual minimum of particle *I* be Pbest, let *ex* = Pbest, *en* = 2pbest, *he* = en/10 in normal cloud computing a (*C* (*ex*, *en*, *he*)), generate a new particle *J* according to the normal cloud generator in Definition 2, and let *I* = *J* to complete the evolution operation.
5. If the iteration limit is reached, the Gbest output will end; otherwise, go to (2).

### 3.3. Analysis of Influence of Parameter Selection on Algorithm Performance

In the mutation operation, select the global extreme value Gbest as *ex*. Because at this time, the algorithm may have fallen into local optimization, and according to the sociological principle, there are often better individuals around the current excellent individuals, so there is more chance to find the optimal solution around them. *en* represents the horizontal width of the cloud. The larger the *en*, the larger the horizontal width and the larger the particle search range. The scope of the search should be expanded in the first stage of evolution, the search accuracy should be improved in the next stage of evolution, and *en* should be reduced dynamically. The global extreme (small) value Gbest of particle evolution gradually approaches the actual extreme value from large to small. In this paper, *en* = 2gbest is taken to realize the dynamic mediation of *en* to a certain extent [21].

It is proportional to the degree of distribution of the cloud droplets. The larger it is, the greater the degree of distribution, and the more the cloud droplets spread. If it is too large, the algorithm loses its stability, and if it is too large, the algorithm loses its stability. The smallness and randomness will be lost to a certain extent. *he* = *en*/10 is taken to mediate the stability of the algorithm.

If the parameter *K* is too large, the mutation will be too high, which will affect the efficiency of the algorithm, and if it is too low, reduce the accuracy of the solution. Also, because the particle herd algorithm has a rapid fusion rate in the first stage of evolution, the fusion rate in the next stage is gradually slowed down, it is difficult to set a completely reasonable fixed value for parameter *k*. In this paper, let *k* = Gbest/2 so that the value of *K* decreases dynamically with the global optimal value Gbest so as to realize adaptive adjustment. To select the change threshold *N*, consider the SpHere function as an example to test the effect of different *N* values on the resolution accuracy of the ICPSO algorithm. The experimental parameters were set as follows: the population size was 100, the initial value range was [−5, 5], the maximum iterative algebra was 1000, and the SpHere function was 5, 10, 30, 50, 100. Take 2 for *N*, respectively. Run 5, 10, and 20 50 times to get the mean, and the quantity is *K* = Gbest/2. For the test results, see Table 1.

As can be seen from Table 1, the smaller the threshold *n* of low-dimensional function with dimension less than 10, the higher the accuracy of the solution, but the more time-consuming. The smaller the threshold *n* of 10∼100-dimensional function, the more time-consuming, but the accuracy of the solution is not necessarily high. There is an inflection point in the solution accuracy at 5 out of *n*. It can be seen that the selection of *n* value has a certain correlation with the dimension of the function [22].

## 4. Result Discussion

Check the effectiveness of the improvement measures, the following typical function extreme value optimization problem is introduced.

(1) RA-Rastrigin function is shown in formula (13):
  (14) $$\begin{array}{c} f_{1}\left(x,y\right)=x^{2}+y^{2}-\cos\;18\;x-\cos\;18\;y, \end{array}$$
where *x*, *y* ∈ [−1,1], the optimization objective is to find the minimum value of the function, the global minimum point of *f*_1_ is (0,0), the global minimum value is −2, and there are about 50 local minimum points in the feasible region. The variation of Rastrigin function optimization results with dimension is shown in Figure 4.
(2) The generalized raster function is shown in equation (14):
  (15) $$\begin{array}{c} f_{2}\left(x\right)=\sum_{i=1}^{30}\left[x_{i}^{2}-10\;\cos\left(2\pi x_{i}\right)+10\right]. \end{array}$$
Here, *x*_*i*_ ∈ [−5.12, 5.12], the optimization objective is to find the minimum of the function, the global minimum of *f*_2_ is 0, and there are about 45 local minimum points in the feasible region.
(3) Br-Branin function is shown in equation (15):
  (16) $$\begin{array}{c} f_{3}\left(x,y\right)={\left(x-\frac{5.1}{4\pi^{2}}y^{2}+\frac{5}{\pi }y-6\right)}^{2}+10\left(1-\frac{1}{8\pi }\right)\cos\;y+10, \end{array}$$
where *X* ∈ [0,15]; *y*∈[−5,10].The optimization objective is to find the minimum of the function, the global minimum of F3 is 0.3979, and the three global minimum points are (−3.031, 1.164), (3.031, 1.164), and (9.3425, 2.425).
(4) The six-hump camel-back function is as follows (16):
  (17) $$\begin{array}{c} f_{4}\left(x,y\right)=4x^{2}-2.1x^{4}+\frac{1}{3}x^{6}+xy-4y^{2}+4y^{4}. \end{array}$$

Here, *x*, *y* ∈ [−5,5], the optimization objective is to find the minimum of the function, the global minimum of F4 is −1.0205, and the two global minimum points are (0.0884, −0.7014) and (−0.0884, 0.7014). The above functions are optimized 50 times with basic CPSO and ICPSO, respectively. For comparison, the initial values of the two algorithms are the same. Then, count the maximum/minimum steps, convergence times, and average steps of each algorithm. The simulation results are shown in Figure 5 ∼ Figure 8 and Table 2.

Figures 5–8 show the comparison curve of CPSO and ICPSO optimization. From the figures, it can be seen that the calculation accuracy of ICPSO is significantly improved and the iteration algebra is reduced. In Figure 5, CPSO does not converge, which verifies the problem of poor optimization ability. After step 10 of ICPSO, it begins to converge stably and gradually approaches the global optimal value −2. In Figures 6 and 7, the curve after CPSO optimization drops relatively slowly, and the speed gradually approaches 0 due to the algorithm itself, and the speed update correspondingly becomes slower and slower. At this time, the particles will gather at several points and cannot conduct larger-scale local search, making the optimization trapped in local convergence. As can be seen from Figure 8, the optimization goal was achieved in step 46, and ICPSO reduced the number of particle iterations and improved the optimization accuracy by transforming the solution space and mutating the normal cloud operator and achieves the optimization goal in step 10 and step 7, respectively. In Figure 8, it can be seen from the optimization curves of CPSO and ICPSO that although the curve change is not very obvious, it is obvious from the number of optimization steps that ICPSO reaches the optimization goal in step 9 and CPSO reaches the optimization goal in step 23. Table 2 shows the performance simulation results of ICPSO combined with two improvement measures and basic CPSO, in which the average number of steps is the average value under convergence. It can be seen from Table 2 that the basic CPSO algorithm within 500 generations has not reached convergence for 8 times, 6 times, 4 times, and 5 times, respectively. In the case of convergence, the average number of steps is much higher than ICPSO, and all the improved algorithms converge. In terms of time performance, the convergence time of ICPSO is much better than that of CPSO algorithm. Comparing the simulation results, the ICPSO algorithm is better than the CPSO algorithm, indicating that the improved method is effective.

## 5. Conclusion

Particle herd optimization is a global research hotspot. Its research includes the analysis of algorithm mechanism, the improvement of algorithm performance and the expansion of algorithm application. CPSO algorithm is based on cloud digital feature coding to better describe the dynamic behavior of cloud particles. Focusing on key CPSO current issues, this paper proposes two improvement measures to improve algorithm search capabilities, population diversity, and algorithm integration speed and accuracy. Experiments have shown that the improved method is effective. The successful combination of cloud model, cloud particle swarm optimization, and mutation idea makes a new exploration and attempt for the research of solving the optimal value. Although some of these issues have been addressed in this paper and some step-by-step results have been achieved, there is still a need for further discussion and in-depth research on some of the issues encountered during the study: Create as many types of problems as possible, or develop algorithms that are more appropriate to the specific situation? There is currently no unified design standard. In this regard, it is necessary to develop a flexible algorithm that can use the properties of the particle herd optimization algorithm for different problems and combine it with the specifics of the problem, and it needs to be adapted.

## Figures and Tables

**Figure 1:** An improved particle swarm optimization algorithm.

**Figure 2:** The schematic diagram of the update process.

**Figure 3:** Cloud model and its digital features.

**Figure 4:** Variation of Rastrigin function optimization results with dimension.

**Figure 5:** RA-Rastrigin function optimization curve.

**Figure 6:** Optimization curve of generalized Rastrigin function.

**Figure 7:** BR-Branin function optimization curve.

**Figure 8:** Optimization curve of six-hump camel-back function.

**Table 1:** Solutions of sphere function under different *N* values.

Dimension	*N* = 2	*N* = 5	*N* = 10	*N* = 20
5	8.674*e* − 154	1.540*e* − 133	4.165*e* − 118	4.555*e* − 110
10	2.868*e* − 118	1.126*e* − 114	4.01*e* − 106	5.200*e* − 100
30	1.081*e* − 056	3.777*e* − 060	1.655*e* − 057	3.058*e* − 050
50	4.100*e* − 038	3.027*e* − 040	3.010*e* − 037	1.080*e* − 030
100	5.016*e* − 018	6.865*e* − 020	4.270*e* − 020	6.071*e* − 015

**Table 2:** Performance comparison between PSO and ICPSO algorithms.

Function	Algorithm	Max/min steps	Average steps	Convergence
RA-Rastrigin	CPSO	500/28	63	41
	ICPSO	28/6	21	49

Generalized Rastrigin	CPSO	500/34	72	43
	ICPSO	34/9	24	49

BR-Branin	CPSO	500/37	67	45
	ICPSO	37/8	20	79

Six-hump camel-back	CPSO	500/27	74	45
	ICPSO	30/6	18	49

## Data Availability

The datasets generated and/or analyzed in the current study are available from the corresponding author upon reasonable request.
